The article "Anti-NMDA Receptor Encephalitis: Retrospective Analysis of 15 Cases, Literature Review, and Implications for Gynecologists" was published in 2022. Journal: J Healthc Eng.

# Anti-NMDA Receptor Encephalitis: Retrospective Analysis of 15 Cases, Literature Review, and Implications for Gynecologists

**DOI:** 10.1155/2022/4299791

**Published:** 2022-03-15

**Authors:** Yibin Liu, Yanpeng Tian, Ruoyi Guo, Xin Xu, Mingle Zhang, Zhongkang Li, Yanlai Xiao, Wen Cao, He Gao, Desheng Kong, Yanfang Du, Li Meng, Jingkun Zhang, Xianghua Huang

**Affiliations:** ^1^Department of Obstetrics and Gynecology, The Second Hospital of Hebei Medical University, Shijiazhuang, Hebei 050000, China; ^2^Department of Neurology, The Second Hospital of Hebei Medical University, Shijiazhuang, Hebei 050000, China

## Abstract

**Background:**

Anti-N-methyl-D-aspartate (NMDA) receptor encephalitis is a rare form of autoimmune encephalitis caused by anti-NMDA receptor antibodies. This disease mainly affects women of childbearing age and is commonly associated with ovarian teratoma. However, the relationship between anti-NMDA receptor encephalitis and ovarian teratoma and the role of anti-NMDA receptor antibody in the relationship remain unclear.

**Objectives:**

This study aimed to describe 15 cases of anti-NMDA receptor encephalitis (5 with ovarian teratoma), review literature, and reinforce the gynecologist's knowledge of this disorder.

**Methods:**

Clinical data of 15 patients from January 2015 to December 2020 admitted to The Second Hospital of Hebei Medical University were collected and analyzed. The diagnosis of anti-NMDA receptor encephalitis was based on the presence of anti-NMDA receptor antibodies in cerebrospinal fluid (CSF) and/or serum. Laparoscopic teratoma removal was performed in patients with ovarian teratoma. All patients had received immunotherapy. In addition, a review of the literature was performed to reinforce the gynecologist's knowledge of this disorder.

**Results:**

A total of 15 patients with anti-NMDA receptor encephalitis were screened, of whom 5 patients were confirmed with ovarian teratoma by pathology. The most common symptoms of anti-NMDAR encephalitis with teratoma are fever (5/5, 100%), seizure (5/5, 100%), mental and behavioral disorders (4/5, 80%), and decreased consciousness (4/5, 80%). Conversely, the most common symptoms of patients without teratoma were neuropsychiatric symptoms, including headache (6/10, 60%) and mental and behavioral disorders (7/10, 70%). All patients underwent immunotherapy, including steroids, intravenous immunoglobulin (IVIG), plasma exchange, and cyclophosphamide, and 4 out of 5 patients with ovarian teratomas underwent surgical treatment. All patients had a good outcome after systemic, surgical, and immunotherapy treatment. No patient who underwent surgical treatment developed a recurrence. Conversely, 2 of 10 patients without teratoma developed an anti-NMDA receptor encephalitis recurrence.

**Conclusions:**

Patients with anti-NMDA encephalitis show severe mental and neurological symptoms. Resection of teratoma is beneficial to the relief or disappearance of symptoms and has a good prognosis. This disorder should be fully recognized by gynecologists, who play an important role in diagnosis and treatment.

## 1. Introduction

In 2005, Vitaliani et al. reported a group of neuropsychiatric symptoms in four young female patients with ovarian teratoma characterized by acute psychiatric symptoms, seizures, memory deficits, decreased level of consciousness, and central hypoventilation [1]. N-methyl-D-aspartate (NMDA) receptor antibodies were subsequently detected in these and other eight female patients with similar symptoms [2]. These findings made it clear that these neuropsychiatric symptoms were mediated by anti-NMDA receptor antibodies. This disorder was then officially named anti-NMDA receptor encephalitis. During the following years, an increasing number of cases were diagnosed as anti-NMDA receptor encephalitis, including children, the elderly, and males [3]. Patients usually presented abnormal behavior, speech dysfunction, movement disorders, decreased level of consciousness, autonomic dysfunction, or central hypoventilation and seizures. Seizures can occur at all stages of this disorder [4]. However, the underlying mechanism of this disease and its relationship with ovarian teratoma are still unclear.

In recent years, a large number of studies indicated that immunosuppressive therapy and teratoma removal are effective treatments for this disorder [5]. Steroids, intravenous immunoglobulin (IVIG), and plasma exchange are first-line immunosuppressive therapies. Patients with a delayed diagnosis or poorly responding to the first-line immunotherapies usually required the second-line immunosuppressive therapies with rituximab and cyclophosphamide. Meanwhile, compared with cases with teratoma after teratoma removal, patients without teratoma often have a poor prognosis. Salome et al. reported a case without teratoma had a good outcome after the removal of normal-appearing ovaries [6]. These findings suggest that the normal-appearing ovary may also play an important role in the disease. Here, we reported 15 cases diagnosed with anti-NMDA receptor encephalitis with or without ovarian teratoma. Clinicopathological features were analyzed and a literature review was performed to systematically analyze the pathogenesis and pathological characteristics of anti-NMDA receptor encephalitis to reinforce the gynecologist's knowledge of this disorder.

## 2. Methods and Materials

### 2.1. Patients

From January 2015 to December 2020, 15 patients diagnosed with anti-NMDA receptor encephalitis were enrolled in this study. All CSF and serum samples from patients with suspected anti-NMDA receptor encephalitis were collected to detect whether the anti-NMDAR antibody was positive. Patients with positive anti-NMDAR antibody in CSF are diagnosed. Details of these patients' clinical information are recorded. The Ethics Committee has approved all the experimental protocols of The Second Hospital of Hebei Medical University. All patients signed the informed consent.

### 2.2. Neurological Examination and Gynecology Evaluation

All patients diagnosed with anti-NMDA receptor encephalitis underwent detailed neurological examination and systematic tumor screening. The imaging examinations comprised brain magnetic resonance imaging (MRI), brain CT, and electroencephalography (EEG). Based on the clinical manifestation of this disease, symptoms were categorized into 6 groups: abnormal (psychiatric) behavior or cognitive dysfunction, speech dysfunction, seizures, movement disorder, decreased level of consciousness, and autonomic dysfunction or central hypoventilation. Pelvic ultrasounds were applied to screen ovarian teratoma.

### 2.3. Treatment

All patients were treated with antiviral and symptomatic therapy before being diagnosed with anti-NMDA receptor encephalitis. Once diagnosed with anti-NMDA receptor encephalitis, all patients received combined immunosuppressive therapy. The first-line immunosuppressive therapy typically consists of steroids, intravenous immunoglobulin (IVIg), and plasma exchange. Upon failure of first-line treatment and/or a delayed diagnosis, second-line immunosuppressive therapy was applied including rituximab or cyclophosphamide alone or in combination. Laparoscopic examination and teratoma removal were performed in patients with ovarian teratoma indicated by pelvic ultrasounds.

### 2.4. Statistical Analysis

Clinical information and symptoms were summarized using descriptive statistics. A Fisher exact test was used to analyze categorical data. Continuous variables were compared by one-way analysis of variance and presented by mean ± SD. Significant differences were set at *P* < 0.05. Statistical analysis was performed with GraphPad Prism 8.0 software.

## 3. Results

### 3.1. Demographics Characteristics of Anti-NMDA Receptor Encephalitis

A total of 15 patients were diagnosed with anti-NMDA receptor encephalitis from 2016 to 2020, of whom 5 were confirmed with ovarian teratoma. The incidence rate of ovarian teratoma was 33.33%. Notably, all patients with teratoma were over 18 years old. The incidence rate of ovarian teratoma was 50% in patients aged >18 years. The average age of all patients was 24.27 ± 9.00 years (range, 15 to 45). The average age of patients with ovarian teratoma was 28.60 ± 3.44 years (range, 24 to 32). The average age of patients without ovarian teratoma was 22.10 ± 10.25 years (range, 15 to 45). Comparisons of clinical features of patients with anti-NMDA receptor encephalitis with or without ovarian teratoma are shown in Table 1.

### 3.2. Clinical Features of Anti-NMDA Receptor Encephalitis

The most common symptoms of anti-NMDAR encephalitis with teratoma are fever (5/5, 100%), seizure (5/5, 100%), mental and behavioral disorders (4/5, 80%), and decreased consciousness (4/5, 80%). However, the incidence rate of fever in patients without teratoma was only 50% (5/10). The most common symptoms of patients without teratoma were neuropsychiatric symptoms, including headache (6/10, 60%) and mental and behavioral disorders (7/10, 70%). All of the five patients with teratoma presented with typical viral-like prodromal symptoms (fever, *T* > 37.5 °C), and two of them also presented with headache. Three of them developed movement disorders and central hypoventilation. In addition, two of them developed autonomic dysfunction (Table 1). However, only half of 10 patients without teratoma presented with typical viral-like prodromal symptoms and seizures. Meanwhile, memory deficit occurred in 2 patients without teratoma, but not in patients with teratoma. Results are shown in Table 1.

Both groups showed slightly different results with regard to comorbidities. Among the 5 patients with teratoma, 2 patients were diagnosed with pulmonary infection and 1 patient with pleural effusion was suspected to be associated with pulmonary infection. Of the 10 patients without teratoma, 2 patients were diagnosed with pulmonary infection, 1 patient was diagnosed with bronchitis, and 1 patient was diagnosed with central nervous system infection. In terms of tumor, 1 patient with teratoma was reported on right breast fibroadenoma and underwent surgical resection, while 1 patient without teratoma was reported on uterine myoma (Table 2).

### 3.3. Laboratory Tests and Diagnosis

All patients underwent MRI, CT, EEG, and anti-NMDA antibody screening. MRI can present with hypersignals in T2/FLAIR sequences in the hippocampus or can be normal. Abnormal EEG was observed in all patients with delta brush or rhythmic delta waves. The diagnosis was confirmed when anti-NMDA receptor antibodies had been detected in CSF and/or serum.

### 3.4. Treatment and Outcome

Of the 5 patients with teratoma, 4 patients underwent surgical treatment and 1 patient refused surgery. Postoperative pathology showed mature cystic teratoma in 3 patients and grade 1 immature teratoma in 1 patient (Figure 1). All patients were treated with first-line immunotherapy and antipsychotic drug therapy, of which 1 patient refused IVIG treatment and another one patient received plasma exchange treatment. In addition, 1 patient received second-line immunotherapy (CTX) treatment. Patients with infections or typical viral-like prodromal symptoms received antibiotics and/or antiviral treatment (Table 3).

All of the 10 patients without teratoma received first-line immunotherapy (glucocorticoids and IVIG) and no patients received second-line immunotherapy. A total of 5 patients were given anti-infection treatment according to flu-like symptoms at the time of admission. Meanwhile, all patients underwent antipsychotic drug therapy.

After 1 month of treatment, all patients' symptoms were relieved. During the 24-month follow-up, all patients had a favorable outcome and there was no death. In addition, no patient who underwent surgical treatment developed a recurrence. Conversely, 2 of 10 patients without teratoma developed an anti-NMDA receptor encephalitis recurrence.

## 4. Discussion

In recent years, anti-NMDA receptor encephalitis has received further attention as a newly identified cause of autoimmune encephalitis. Although studies have shown the important role of anti-NMDA receptor antibodies in the disease, the pathogenesis is still not clear [2, 3]. Based on a review of the literature and clinicopathological features of the 15 cases in our series, we attempted to summarize the pathogenesis, clinical features, diagnosis, treatment, and latest research advances.

### 4.1. Structure and Function of NMDA Receptor

NMDA receptor is a subtype of ionotropic glutamate receptors regulating excitatory synaptic transmission in the central nervous system (CNS), which is involved in multiple physiological and pathological processes, such as learning, memory, drug addiction, and neurodegenerative diseases[7–9]. Functional NMDA receptors are heteromeric complexes composed of two GluN1 subunits together with either two GluN2 subunits or a combination of GluN2 and GluN3 subunits[10, 11]. GluN1 and GluN3 subunits provide glycine binding sites, whereas GluN2 subunits bind glutamate [12]. When excitatory neurotransmitters, such as glutamate, were released from presynaptic neurons to act on the AMPA receptor of the postsynaptic membrane, the AMPA receptor is activated and a large amount of sodium ion flows in, causing the depolarization of postsynaptic neurons. When the neurons depolarize to a potential level of −50 mV or more positive, the blocking effect of Mg^2+^ on the NMDA receptor is lifted, and a large amount of calcium ions flow into the cell through the NMDA receptor, triggering long-term potentiation in postsynaptic neurons [13–15]. In addition, Ca^2+^, as an important second messenger in the cell, activates a series of signaling pathways to play a biological regulatory role. Therefore, abnormal expression and function of NMDA receptors can cause disorders of central nervous system function.

### 4.2. Epidemiology

Since anti-NMDA receptor encephalitis was first reported and named by Dalmau et al., thousands of cases have been identified [1, 2]. Unlike the earliest discovery that this disease was associated with teratoma, female youth without teratoma and even male and children patients were also reported in subsequent studies [3]. Titulaer et al. reported 577 patients with anti-NMDA receptor encephalitis [16]. The results showed that the disease can occur at any age in the life cycle, with a peak age of onset between 12 and 45 years in females. Among patients younger than 12 years and older than 45 years, the proportion of males can account for 40%. Thirty-eight percent of the patients had tumors, 97% of those with tumors were women, and 96% of the tumors were ovarian teratomas. Extraovarian teratomas, lung cancer, breast cancer, testicular cancer, ovarian cancer, thymic cancer, and pancreatic cancer have also been successively found in patients with anti-NMDA receptor encephalitis, but the relationship between these tumors and this disease still needs further investigation [16]. Dai et al. reported 108 female patients with anti-NMDA receptor encephalitis, which is by far the largest single-center prospective study in mainland China [17]. These results showed 29 patients (26.9%) were confirmed with ovarian teratoma by pathology. In our study, 5 out of 15 patients (33.3%) were confirmed with ovarian teratoma, which is consistent with findings in previous studies.

### 4.3. Pathogenesis

Recent studies suggest that the Fc segment of the anti-NMDA receptor IgG antibody mediates the binding, cross-linking, capping, and reversible internalization of NMDA receptors, and loss of NMDA receptors from synaptic and extrasynaptic space correlates with antibody titer [18]. In addition, incubating hippocampal neurons with the patient's CSF or purified IgG antibody caused the internalization of NMDA receptors and the reduction of synaptic NMDA receptor-mediated currents [18, 19]. In contrast to these effects on NMDA receptors, patients' antibodies did not alter the localization or expression of other glutamate receptors, the number of synapses, dendritic spines, dendritic complexity, or neuron survival. Studies have pointed out that the reduction of NMDA receptors could cause excessive accumulation of glutamates, and the accumulated glutamates act on NMDA receptors to induce excessive activation, resulting in excitotoxicity caused by intracellular calcium overload [20]. It might be the underlying mechanism of seizures. However, more studies are needed to confirm whether the conjecture is correct. In Day et al.'s study, abnormal neuroglial elements were found in teratomas resected from patients with anti-NMDA receptor encephalitis but not in teratomas from controls without neurological dysfunction [21]. These results demonstrated that abnormal neuron components and inflammatory infiltrates within teratomas resected from patients with NMDA receptor encephalitis might be the basis of the selective immune response characteristic of teratoma-related diseases. Moreover, Salome et al. reported a case with normal ovary had a good outcome after a bilateral salpingo-oophorectomy after the failure of conservative immunotherapy [6]. These results indicated that normal ovaries might also play a critical role in the initiation and progression of anti-NMDA receptor encephalitis. Tachibana et al. study found NMDA receptors were expressed in the bovine ovum [22]. This study further confirmed that normal ovaries might play a role in this disease. Although current studies have shown that anti-NMDA receptor antibodies are the main factor in the disease, the mechanisms of autoantibody production, the relationship between antibodies and ovarian teratomas, and how the antibodies cross the blood-brain barrier are still unclear.

### 4.4. Clinical Features

According to the disease natural progression, the clinical course exhibited five phases: the prodromal phase, the psychotic phase, the unresponsive phase, the hyperkinetic phase, and the gradual recovery phase [23]. In the prodromal phase, most patients will have nonspecific flu symptoms lasting five to fourteen days, such as fever, headache, shivering, nausea, and vomiting [24, 25]. In hospital visits during this phase, patients are often misdiagnosed with acute upper respiratory tract infection or influenza. Patients subsequently developed a range of neuropsychiatric symptoms and behavioral disturbances. Apathy, fear, depression, impaired cognitive skills, psychosis, and seizures are the primary clinical symptoms [26, 27]. Generalized tonic-clonic is the most common seizure pattern [28]. Patients are often referred for psychiatric assessment and may be treated with psychoactive agents, psychotherapy, or admission to the department of psychiatry in this psychotic phase. In addition, some of the patients may be diagnosed with influenza-related encephalitis. In the unresponsive phase, patients were unresponsive to verbal commands, pain, and visual threats. Bizarre and inappropriate smiling can be presented [23, 29]. There was no discernible boundary between the psychotic phase and the unresponsive phase [30]. In the hyperkinetic phase, patients are also characterized by involuntary orofacial movements and dysautonomia manifesting with grimace, chewing behaviors, clenching of teeth, cardiac arrhythmia, labile blood pressure, and hypoventilation [23, 27]. After teratoma removal and immunosuppressive therapy, patients will develop into gradual recovery phase. All symptoms were gradually relieved. However, not all patients experienced all these stages. According to its clinical presentation, Titulaer et al. summarized 8 groups of symptoms: behavior and cognition disturbance, memory deficit, speech impairment, seizures, movement disorder, loss of consciousness, autonomic dysfunction, and central hypoventilation [16]. Movement disorders are more common in children, while memory deficits and central hypoventilation are more common in adults.

### 4.5. Diagnosis

Due to the lack of specific symptoms, it is difficult to diagnose at early stage and there are no specific findings in MRI. Some patients can exhibit hypersignals in T2/FLAIR sequences in a variety of regions (hippocampus, cortex, cerebellar, and brainstem) [2, 16, 31]. The most accurate diagnostic method for anti-NMDA receptor encephalitis is the positivity of the anti-NMDA antibodies in the serum and/or CSF [32]. Dalmau recommends the positivity of the anti-NMDA antibodies in both the serum and CSF [24], whereas Irani and Vincent indicate the antibody titer in serum was higher than that in CSF [33]. To more precisely diagnose early stages, diagnostic criteria for anti-NMDA receptor encephalitis were published in 2016 [4]. The criteria are shown in Table 4 [4, 34]. In addition, routine screening for ovarian teratoma is necessary for all female patients.

### 4.6. Treatment and Outcome

The treatment principles of anti-NMDA receptor encephalitis are etiology, immunotherapy, symptomatic therapy, and supportive treatment. For those patients with teratomas, surgical treatment is still a particularly important procedure. Previous studies have indicated early surgical resection of ovarian teratomas can significantly improve neuropsychiatric signs and decrease relapse [35]. Florance et al. reported that complete recovery occurred more frequently in patients (5/8, 62.5%) with ovarian teratoma removal than in those (4/23, 17.39%) without ovarian teratomas [28]. Therefore, it should be noted that ovarian teratomas should be resected once detected and severe neuropsychiatric symptoms should not be contraindications for surgery [17, 36]. Moreover, the same recommendations apply to patients during pregnancy [37]. In our studies, 4 out of 5 patients underwent surgery. For those without ovarian teratomas, immunosuppressive therapy is an effective regimen. Corticosteroids, intravenous immunoglobulins, and plasma exchange are the first-line therapeutic strategies for anti-NMDA receptor encephalitis in combination or alone. When the first-line therapies failed, rituximab and/or cyclophosphamide were recommended as second-line therapies [5]. Patients in severe condition frequently require supportive therapies, including vital sign monitoring, antipsychotics, antiepileptics, mechanical ventilation, and trophic support. After systemic immunotherapy, approximately 75% of patients could recover or have mild sequelae [3, 31]. Meanwhile, ovarian teratoma removal was associated with a 23% reduction in the risk of relapse [17].

### 4.7. Prospects and Challenge

Here, we reported 15 cases with anti-NMDA receptor encephalitis, including 5 patients with ovarian teratomas. All patients have a good outcome after ovarian teratoma removal and immunotherapy. However, there are still some patients with poor response to treatment [3]. In addition, the underlying mechanisms for those without ovarian teratomas are still not fully understood. Although previous studies have shown that the removal of normal ovarian tissue confirmed by pathology is beneficial to the patients' rehabilitation, it is still unclear whether normal ovaries play a potential role in the disease [6]. Is it possible to envisage bilateral oophorectomy for patients whose imaging examination shows no ovarian teratomas? It is needed to weigh the benefits expected from a bilateral oophorectomy and the detrimental effects on the reproductive function [32].

## 5. Conclusion

Anti-NMDA receptor encephalitis, as severe autoimmune encephalitis, should be paid full attention by gynecologists.

## Figures and Tables

**Figure 1:** Ovarian teratomas removed from patients. (a–c) Case 2 from Table 3. (d) Case 3 from Table 3.

**Table 1:** The clinical features of anti-NMDA receptor encephalitis with or without ovarian teratoma.

Variables	Anti-NMDA receptor encephalitis with ovarian teratoma (*n* = 5)	Anti-NMDA receptor encephalitis without ovarian teratoma (*n* = 10)
Age (years)	28.60 ± 3.44 (range, 24–32)	22.10 ± 10.25 (range, 15 to 45)
<18	0	6
≥18	5	4
Fever (*T* > 37.5 °C)	5/5, 100%	5/10, 50%
Headache	2/5, 40%	6/10, 60%
Mental and behavioral disorders	4/5, 80%	7/10, 70%
Speech dysfunction	1/5, 20%	2/10, 20%
Movement disorders	3/5, 60%	3/10, 30%
Decreased consciousness	4/5, 80%	3/10, 30%
Seizure	5/5, 100%	5/10, 50%
Central hypoventilation	3/5, 60%	1/10, 10%
Autonomic dysfunction	2/5, 40%	4/10, 40%
Memory deficit	0/5, 0%	2/10, 20%

**Table 2:** Complications of patients with or without ovarian teratoma.

No.	A	T	Complications		
1	16	No	No		
2	17	No	Pulmonary infection	Hypokalemia	
3	16	No	Hypokalemia		
4	22	No	Right ovarian cysts		
5	45	No	Uterine myoma	Bronchitis	
6	22	No	No		
7	36	No	No		
8	15	No	Subclinical hyperthyroidism	Hyperhomocysteinemia	
9	17	No	Pulmonary infection		
10	15	No	Central nervous system infection		
11	26	Yes	Postoperative of right breast fibroadenoma	Hypoproteinemia	Hypofibrinogenemia
12	31	Yes	Pulmonary infection		
13	32	Yes	Pulmonary infection		
14	24	Yes	Liver dysfunction		
15	30	Yes	Small bowel obstruction	Pleural effusion	

A: age; T: tumor (ovarian teratoma).

**Table 3:** Clinical features and treatment for 5 patients with ovarian teratoma.

No.	Age	Ovarian teratoma	Surgery				Treatment							
		Side	Surgical treatment	Operative pathway	Surgical procedure	Pathology	First-line therapy			Second-line therapy		Other treatments		
							Glucocorticoid	IVIG	Plasma exchange	Rituximab	CTX	Antibiotics	Antiviral drug	Antipsychotic drug
1	26	Left ovary	Yes	Laparoscopic	Laparoscopic ovarian cyst excision	Immature teratoma grade 1	Yes	Yes	Yes	No	No	Yes	No	Yes
2	31	Right ovary	Yes	Laparoscopic	Laparoscopic adnexectomy	Mature cystic teratoma	Yes	Yes	No	No	No	Yes	Ys\es	Yes
3	32	Left ovary	Yes	Laparoscopic	Laparoscopic ovarian teratoma excision	Mature cystic teratoma	Yes	Yes	No	No	Yes	Yes	Yes	Yes
4	24	Left ovary	No	—	—	—	Yes	No	No	No	No	No	Yes	Yes
5	30	Bilateral ovaries	Yes	Laparoscopic	Laparoscopic ovarian teratoma excision	Mature cystic teratoma	Yes	Yes	No	No	No	Yes	Yes	Yes

**Table 4:** Diagnostic criteria for anti-NMDA receptor encephalitis.

Probable anti-NMDA receptor encephalitis
Diagnosis can be made when all three of the following criteria have been met
(1) Rapid onset (less than 3 months) of at least four of the six following major groups of symptoms
Abnormal (psychiatric) behavior or cognitive dysfunction
Speech dysfunction (pressured speech, verbal reduction, mutism)
Seizures
Movement disorder, dyskinesias, or rigidity/abnormal postures
Decreased level of consciousness
Autonomic dysfunction or central hypoventilation
(2) At least one of the following laboratory study results
Abnormal EEG (focal or diffuse slow or disorganised activity, epileptic activity, or extreme delta brush)
CSF with pleocytosis or oligoclonal bands
(3) Reasonable exclusion of other disorders (appendix)
Diagnosis can also be made in the presence of three of the above groups of symptoms accompanied by a systemic teratoma
Exclusion of recent history of herpes simplex virus encephalitis or Japanese B encephalitis, which might result in relapsing immune-mediated neurological symptoms
Definite anti-NMDA receptor encephalitis
One or more of the six major groups of symptoms and IgG GluN1 antibodies (antibody testing should include CSF); if only serum is available, confirmatory tests should be included (e.g., live neurons or tissue immunohistochemistry, in addition to a cell-based assay)
Exclusion of recent history of herpes simplex virus encephalitis or Japanese B encephalitis, which might result in relapsing immune-mediated neurological symptoms

[4, 34]

## Data Availability

The analysed datasets generated during the study are available from the corresponding author on reasonable request.
